# Mesenchymal stem cell derived hematopoietic cells are permissive to HIV-1 infection

**DOI:** 10.1186/1742-4690-8-3

**Published:** 2011-01-12

**Authors:** Timo Z Nazari-Shafti, Eva Freisinger, Upal Roy, Christine T Bulot, Christiane Senst, Charles L Dupin, Abigail E Chaffin, Sudesh K Srivastava, Debasis Mondal, Eckhard U Alt, Reza Izadpanah

**Affiliations:** 1 Applied Stem Cell Laboratory, Heart and Vascular Institute, Department of Medicine, Tulane University Health Science Center; New Orleans, Louisiana, USA; 2 Department of Pharmacology, Tulane University Health Sciences Center, New Orleans, Louisiana, USA; 3 Department of Surgery, Tulane University Health Science Center; New Orleans, Louisiana, USA; 4 Department of Biostatistics, Tulane University School of Public Health and Tropical Medicine, New Orleans, LA, USA; 5 Division of Plastic and Reconstructive Surgery, Louisiana Health Sciences Center, Louisiana State University; New Orleans, Louisiana, USA

## Abstract

**Background:**

Tissue resident mesenchymal stem cells (MSCs) are multipotent, self-renewing cells known for their differentiation potential into cells of mesenchymal lineage. The ability of single cell clones isolated from adipose tissue resident MSCs (ASCs) to differentiate into cells of hematopoietic lineage has been previously demonstrated. In the present study, we investigated if the hematopoietic differentiated (HD) cells derived from ASCs could productively be infected with HIV-1.

**Results:**

HD cells were generated by differentiating clonally expanded cultures of adherent subsets of ASCs (CD90^+^, CD105^+^, CD45^-^, and CD34^-^). Transcriptome analysis revealed that HD cells acquire a number of elements that increase their susceptibility for HIV-1 infection, including HIV-1 receptor/co-receptor and other key cellular cofactors. HIV-1 infected HD cells (HD-HIV) showed elevated p24 protein and *gag *and *tat *gene expression, implying a high and productive infection. HD-HIV cells showed decreased *CD4*, but significant increase in the expression of *CCR5*, *CXCR4*, *Nef*-associated factor *HCK*, and *Vpu*-associated factor *BTRC*. HIV-1 restricting factors like APOBEC3F and TRIM5 also showed up regulation. HIV-1 infection increased apoptosis and cell cycle regulatory genes in HD cells. Although undifferentiated ASCs failed to show productive infection, HIV-1 exposure increased the expression of several hematopoietic lineage associated genes such as *c-Kit*, *MMD2*, and *IL-10*.

**Conclusions:**

Considering the presence of profuse amounts of ASCs in different tissues, these findings suggest the possible role that could be played by HD cells derived from ASCs in HIV-1 infection. The undifferentiated ASCs were non-permissive to HIV-1 infection; however, HIV-1 exposure increased the expression of some hematopoietic lineage related genes. The findings relate the importance of ASCs in HIV-1 research and facilitate the understanding of the disease process and management strategies.

## Background

Human immunodeficiency virus type 1 (HIV-1), the etiologic agent of acquired immune deficiency syndrome (AIDS), predominantly infects hematopoietic cells such as T-helper lymphocytes, monocytes and macrophages. Despite the development of highly active anti-retroviral therapy (HAART), the persistence of reservoirs of HIV-1 poses obstacles to the eradication of the disease. Although initial viral decay kinetics in plasma had indicated optimistic outcomes of HAART [1], long-term measurements have suggested that mononuclear lymphocytes harbor the virus for prolonged periods of time [2].

Infection of lymphoid and myeloid lineages is mediated by recognition of the T-cell receptor CD4 or by the chemokine co-receptors CXCR4 and CCR5. CXCR4 appears to be the most important for HIV-1 entry into T-lymphocytes (T-tropic), whereas CCR5 is known for viral entry into cells such as monocytes and macrophages (M-tropic) [3]. These receptors promote viral attachment and fusion to cellular membranes, thus facilitating entry into hematopoietic cells [4]. Although the peripheral blood-derived hematopoietic progenitor cells (HPCs) can express the HIV-1 co-receptors [5], susceptibility to either T-tropic or M-tropic strains of HIV-1 seem to correlate only with lineage commitment of HPCs [6]. Even though an early loss of circulating CD34^+ ^HPCs and impaired clonogenic potential and apoptosis of these progenitor cells have been documented in HIV-1 infected individuals [7,8], the evidence of productive infection of HPCs remains controversial [9,10].

The mesenchymal stem cells (MSCs) are endowed with multi lineage differentiation potentials and self-renewal properties, which qualify them as potential sources for cell transplantation and gene therapy. MSCs from several origins, including bone marrow and adipose tissue, have been well described. Adipose tissue derived MSCs (ASCs), like bone marrow derived MSCs, have the capacity to differentiate along multiple lineages at clonal levels. They can differentiate into neurons, cardiomyocytes, chondrocytes, osteocytes, and adipocytes [11-16]. However, it is not known whether lineage specific differentiation of MSCs would enable them to be infected by HIV-1 and whether they may act as long-term viral reservoirs within systemic sites.

The HIV-1 infection of bone marrow mesenchymal progenitors and of mesenchyme-derived cells (e.g., fibroblasts and endothelial cells) present in various peripheral organs has been shown to occur via both M-tropic and T-tropic strains of HIV-1 [17-19]; however, integrated provirus is rarely found in these cells and a productive infection has not been documented. However, *in vitro *infection of stromal cells grown in long-term bone marrow cultures (LTBMC) with HIV-1 has been reported [20-22]. Our previous studies had shown that a T-tropic strain of HIV-1 can infect bone marrow MSC cultures and decrease their colony forming ability and adipogenic potential [23]. Further, it has also been shown that multipotent human progenitor cells isolated from fetal brains are permissive towards HIV-1 infection [24]. However, it has not been well established as to how these mesenchyme derived cells become susceptible to HIV-1 and whether their HIV-1 production rates are comparable to that observed in HIV-1 infected lymphoid or myeloid cells. Importantly, despite the possible presence of ASCs in systemic organs, there is no evidence about the ability of HIV-1 to infect either undifferentiated ASCs or their differentiated counterparts.

Recent work from our laboratory has demonstrated that under specific *in vitro *stimulations even the CD34^- ^ASC clones (CD90^+^, CD105^+^, CD45^- ^and CD34^-^) could undergo hematopoietic differentiation (HD) and display macrophage-like characteristics [25]. Macrophages are known to play a crucial role in both HIV-1 infectivity and pathogenesis. Although they can generate high levels of viral progeny, they are resistant to HIV-1 induced cytopathic effects and harbor the virus for a long time [26-28]. Hence, our efforts were focused on studying the susceptibility of the ASCs and the HD-differentiated ASCs for HIV-1 infection and their subsequent abilities to support viral replication. Initially, the differentiated cells were analyzed for receptors, ligand binding, and cofactors, which are directly involved in HIV-1 infection, followed by analysis of changes in gene expression that occurs following HIV-1 infection. Both HIV-1 susceptibility markers and productive replication in HIV-1 exposed HD cells were compared with those observed in a HIV-1 infected T-cell line, and the findings are reported in the present study.

## Results

### Up-regulation of HIV-1 susceptibility genes in HD cells

HD cells were prepared by differentiating expanded cultures of ASC clones, phenotypically identified as CD90^+^, CD105^+^, CD44^+^, CD4^-^, CD68^-^, CD34^-^, CD45^-^, and CD11b^- ^cells as described previously [25]. For the initial assessment of HD cells, we performed a transcriptomic analysis after 8 days of differentiation. The HD cells expressed a number of HIV-1 receptors such *CD4 *(33.9 ± 3.4 fold), *CXCR4 *(2.7 ± 0.42 fold), *CCR4 *(1.64 ± 0.05 fold), and *CCR5 *(1.93 ± 0.26 fold) compared to undifferentiated ASCs (Figure 1A). HD cells also expressed a series of genes involved in innate and adaptive immune reactions and key cellular cofactors for HIV-1 infection such as *IL-8*, *SERPINA1*, *CCL8*, *CD69 *and interleukins 2, 10, and 16 (Figure 1B). The expression of lymphoid associated gene *BCL11B *was markedly up regulated. Further, the expression of a number of cell cycle regulators, such as *BAX*, *CDKN1A*, *FOS*, *GADD45A*, *NFATC1*, *CEBPB*, *STAT1*, and *STAT3*, decreased while the expression of *NFκB1A *slightly increased as a result of differentiation (Figure 1C).

**Figure 1:** **Gene expression analysis of HD cells following hematopoietic differentiation**. Compared to ASCs, the expression level of HIV receptor genes (*CD4, CXCR4, CCR4*, and *CCR5*) were up regulated in HD cells as result of differentiation **(A)**. Expression of several genes involved in innate and adaptive immune reactions **(B)**, and cell cycle regulators **(C) **were altered in HD cells. A fold change was applied to select genes (P < 0.05). All values are normalized to ASCs (X axis).

### A highly productive HIV-1 infection is evident in virus exposed HD cells

Since cells of the hematopoietic system are among the main targets of the HIV-1 virus, we investigated the effect of viral exposure on HD cells. Clonally expanded cells were allowed to differentiate into HD cells for 5 (5-HD) or 8 (8-HD) days in differentiation media. For analyzing the infectivity of HD cells, we exposed them to very low levels of HIV-1 virus (10^3^-10^4 ^TU/10^5 ^cells or 0.1 MOI) for 24 hours. Unbound viral particles were removed and cultures maintained for an additional 5 days. Following infection of HD cells, noticeable morphological changes beginning from day 3 post-infection were observed. These morphological changes heralded a loss of significant numbers of cells by day 5 post-infection, indicating the dominance of viral infection on HD cells (Figure 2). Subsequently using ELISA for HIV-1 p24, we assayed the levels of HIV-1 p24 released in the supernatant of HD-HIV, and HIV-1 exposed undifferentiated ASCs (ASCs-HIV) cultures which served as controls. The concentration of p24 in culture supernatant is depicted in Figure 3A.

**Figure 2:** **Morphological changes in differentiated HD cells following exposure to HIV-1**. Day-0, HD cells which are on day 8^th ^of differentiation and before viral infection. Day-3, shows the morphological changes of HD cells following 72 hours of viral infection. Day-5, morphology of HD cells infected with HIV-1 virus following 120 hours of infection. Images were taken with Nikon Eclipse 2000. Scale bar is 100 μm.

**Figure 3:** **Expression of HIV-1 p24 protein in HD-HIV and ASC-HIV cells.** p24 antigen level was monitored following post exposure to HIV-1 for 24 hr. HIV-1 was exposed to undifferentiated, 5-HD and 8-HD cells and p24 level was measured after 1, 3 and 5 days following removal of virus **(A)**. Data represent the compilation of three separate experiments carried out in triplicates (P < 0.0001). **(B)** HIV-1 *gag *expression in HD-HIV and HUT78-HIV cells and compared to HIV-1 exposed ASCs (P < 0.05). **(C)** mRNA was extracted from ASC-HIV, HD-HIV, and HUT78-HIV cells and RT-PCR was performed for *Tat *expression.

Both 5-HD and 8-HD cultures showed consecutively increasing levels of p24 on days 3 to 5. On day 5 of infection, p24 levels in 5-HD and 8-HD cultures remained unchanged; the p24 levels in ASCs-HIV were negligible, indicating no evidence of viral replication.

To quantify HIV-1 cDNA and proviral DNA, the mRNA level of "*gag*" and "*Tat*" were assayed. Figure 3B shows the increased expression of *gag *in HD-HIV cells 3 days post infection. This level decreased significantly by day 5 after infection. The *gag *expression in HD-HIV cells was comparable to the HIV-1 infected "HUT-78" (HUT78-HIV), a T-lymphoblastoid cell line that served as a positive control in these experiments. The RT-PCR experiments showed enhanced expression of *Tat *in HD-HIV and HUT78-HIV cells (Figure 3C). The expression of *gag *and *Tat *were not detected in ASCs-HIV.

### HIV-1 infection significantly alters the gene expression profile in HD cells

The expression of selected genes mainly involved in HIV-1 infection and immune response was analyzed as described in the methods. The results obtained for each group, normalized to the mean value of the house keeping gene, were compared by scatter plot analysis using PCR-array data analysis software (SABiosciences). To study the effect of viral exposure on HD cells, we compared the expression of selected genes in HD-HIV cells versus un-infected HD cells. The gene profile of HD-HIV cells was then compared to HUT78-HIV cells. The analysis showed that HIV-1 infection altered gene expression within HD cells in a similar fashion to that seen in HUT78-HIV cells. Several genes were perturbed in response to viral exposure, and these included genes coding for HIV-1 receptors and ligands (*CCL4, CCL5, CCR5, CXCL12, CXCR4, CXCL12*). The viral exposure showed its maximum effect on the HD-HIV cells, when compared to HUT78-HIV cells (Figure 4A).

**Figure 4:** **Comparison of the gene expression profiles of HIV-1 infected HD and HUT78 cells**. Genes that were found to be differentially expressed in HD-HIV vs. HD cells in one set and HD-HIV vs. HUT78-HIV cells in another set were then grouped according to functional categories including genes encoding for HIV-1 receptors and ligands (A), cell cycle and apopotosis (B), and cellular factors involved in HIV-1 infection (C). A fold change was applied to select genes (P < 0.05). All values are normalized to either ASCs or HD cells (X axis).

HIV-1 infection also profoundly altered expression of the cell cycle and apoptosis regulatory genes including *BAX, BCL2, CDKN1A, GADD45A, CDk9, IRF1, CEBPB*, and *IRF2*. The changes in the expression levels of these genes were more pronounced in HD-HIV cells when compared to HUT78-HIV. However, there were smaller differences in the expression levels of *Caspase 3, NFκBIA, TNSF10, STAT1*, and *STAT3 *(Figure 4B).

HIV-1 infection caused significant changes in the expression of cellular factors involved in HIV-1 infection such as *BANF1, CD247, TRIM5, VPS4A, XPO1, CD209 *and to a lesser extent, changed the expression levels of a β-transducin repeat containing (*BTRC*), *CBX5*, and *HTATSF1*. HD cells showed enhanced expression of genes coding for factors known to restrict HIV-1 replication such as *CD209, APOBEC3F*, Tat specific factor 1 (*TAT-SF1*), and tripartite motif-containing 5 (*TRIM5*) (Figure 4C).

Immunocytochemistry was employed to analyze the expression of CCR4, CCR5, NOS2 and CXCR4 proteins in HD-HIV cells. As shown in Figure 5, these markers could be readily detected in approximately all cells. However, the expression of CD4 was in undetectable levels by immunohistochemistry

**Figure 5:** **Expression of hematopoietic markers in HD cells following HIV infection**. Immunohistochemistry of HD-HIV cells, fluorescent images indicate the expression of CCR5, CCR4, NOS2, and CXCR4. Right panel shows the DIC images of identical fields. Images were obtained with Leica TCS SP-2 confocal microscope. Scale bar 10 μm.

### Productive infection is not seen in undifferentiated ASCs

Undifferentiated ASCs exposed to HIV-1 resulted in no significant productive infection up to 5 days. In addition, viral exposure did not cause noticeable effects on the viability of ASCs. Exposure to low MOI (0.1) of the virus did not show any significant effect on the expression of *CD4, CD14, CD68, MSR1, TNFα *and *MRC1 *in ASCs. However, exposure to HIV-1 resulted in a provisional up-regulation of *c-Kit *(6.4 ± 1.4 fold, p ≤ 0.05), *IL10 *(188.9 ± 1.6 fold, p ≤ 0.01) and *MMD2 *(65 ± 1.1 fold, p ≤ 0.01) by day 3 post-exposure. By day 5, the expression of these genes decreased, however, the levels were still higher than in the un-exposed control ASCs (*IL10 *= 67.5 ± 1.5, p ≤ 0.01; *MMD2 *= 24.3 ± 1.3, p ≤ 0.01; and *c-Kit *= 4.1 ± 1.9, p ≥ 0.05). The decline in the expression of *MMD2 *on day 5 as compared to day 3 was significant (p ≤ 0.01) (Figure 6). Our observations indicate that the HIV-1 exposed ASCs showed significantly lower adipogenic, osteogenic potential. However, HIV exposure seems to expedite the generation of HD cells to less than 5 days (from the normal 8 days), when placed in hematopoietic differentiation media. The generated HD cells from HIV-1 exposed ASCs did not exhibit any evidence of productive infection.

**Figure 6:** **Effects of HIV-1 exposure on gene expression of ASCs**. The gene expression levels were calculated based on the dCT-values which have been standardized with the GADPH levels. The ASCs (n = 4 donors) were harvested following 3 and 5 days after exposure to HIV-1. *IL10*, *c-Kit*, and *MMD2 *expression increased significantly by 3 days post HIV-1 exposure (P < 0.05, * represents P < 0.01). The ASCs showed no morphological changes during the course of experiment.

The possible integration of HIV-1 in an exposed ASC genome was examined by repetitive-sampling *Alu-gag *PCR technique described earlier [29]. Briefly, on a nested based PCR technique, the regions of varying length between genomic *Alu *repeats and the HIV *gag *were amplified from the DNA of exposed ASCs to 0.1 MOI of HIV-1 for 24 h. Following this, the second PCR was performed on specific regions of the HIV-1 genome. No evidence of HIV-1 integration was observed in exposed ASCs.

## Discussion

In postnatal and adult life, macrophages differentiate from progenitor cells through various pathways. Macrophages are known to be one of the most important targets for HIV-1 infection and play a crucial role in both viral latency and recrudescence. The CD34^+ ^hematopoietic progenitor cells are commonly known to generate macrophages. Furthermore, the ability of embryonic stem cells to generate HIV-1 susceptible macrophages has been reported [30]. For the first time we showed that a clonally expanded CD90^+^, CD105^+^, CD44^+^, CD4^-^, CD34^-^, CD45^-^, CD11b^-^, CD68^- ^subset of ASCs could also generate cells with macrophage attributes [25]. In the present study, we show that the generated HD cells support productive HIV-1 infection. We show the expression of several HIV-1 susceptibility genes as well as several immune response genes in HD cells. A number of such newly expressed genes may possibly be involved in increasing the susceptibility of HD cells to HIV-1 infection.

Previously we showed that early in differentiation, HD cells develop CD4, a T-lymphocyte marker [25]. Since we utilized the HTLV-III_B _strain which is a T-tropic virus, the infectivity in HD cells as compared to the newly infected HUT78 cells can be explained by utilizing CD4 as one of the most important HIV-1 receptors. Furthermore, as a result of differentiation, expression of other common cellular ligands essential for HIV-1 infection, such as *CXCR4, CCR4*, and *CCR5*, distinctly increased. In addition, the expression of markers associated with activated immune cells, such as the serine protease inhibitor *SERPIN-A1*; the cell surface markers such as *CCL8, CD69*; as well as the expression of interleukins such as *IL-2, IL-8, IL-10*, and *IL-16*, were markedly increased in the HD cells. These observations clearly indicated that these mesenchymal origin cells acquired the attributes of hematopoietic cells.

Our current findings clearly demonstrate a profound increase in the susceptibility of HD cells to HIV-1 infection. Interestingly, higher levels of p24 expression were observed in 8-HD compared to 5-HD cells. This is suggestive that 8-HD cells develop even more cellular receptors for viral entry and are prone for replication. The negligible amount of p24 in ASCs-HIV might be associated with a residual amount of virus floating in the media. Compared to HUT78 cells, the HD cells supported a highly productive HIV-1 infection as evident from the significantly higher levels of *gag *and *Tat *expression in both cell types post HIV-1 exposure. The *gag *expression level decreased in HD-HIV on day-5 post infection which was due to considerable cytotoxicity associated with the HIV infection (Figure 3B).

In order to demonstrate the infectivity of HD cells, we exposed them to very low levels of the virus (0.1 MOI). Indeed, similar to the high level of infectivity observed in the HUT78 cells, the HD cells showed increasing levels of p24 in the supernatants on both day-3 and day-5 post infection, suggesting a possible and crucial role *in vivo *in providing infectable cells.

Interestingly, HIV-1 exposed cells showed a significant decrease in expression of *CD4*. Significant increases in the expression of HIV-1 co-receptors, both CCR5, and CXCR4 were observed in the HD-HIV cells in both gene and protein levels. Although we have not carried out studies using an M-tropic virus, our findings point towards virus infection that enables HD cells to be susceptible to both of R5 and X4 viruses. Previous reports determined that the HIV-1 Tat protein alters co-receptor expression in lymphoid and myeloid cells [31,32]. Studies from our laboratory on the HPC cell line, K562 had also indicated that Tat can differentially regulate both CXCR4 and CCR5 expression in erythroid or megakaryocytic cells [33]. Although we have not measured Tat expression in the HD-HIV cells, the level of productive infection clearly suggests high levels of Tat protein which may be directly involved in changes in HIV-1 receptor expression observed in these cells.

As compared to the newly infected HUT78-HIV cells, the HD-HIV cells showed significantly higher level of expression of several chemokines such as *CXCL12*, *CCL4 *and *CCL5*. CCL4 (MIP-1β) is a major HIV-suppressive factor produced by CD8^+ ^T cells [34]. It has also been documented that MIP-1α and RANTES, as ligands for CCR5, may suppress HIV-1 infection as well [35]. An increase in CXCL12 (SDF-1α) in lymphocytes has also been associated with decreased infectivity of HPCs via the X4-tropic strains of HIV-1 [32]. In HD-HIV cells, the increased expression of several chemokines may thus suggest that the cells are combating to inhibit virus infection by producing these ligands which compete for HIV-1 binding to cells. In addition, this may also suggest that by secreting these chemokines the HD-HIV cells may enhance the recruitment of virus infectable cells to the microenvironments *in vivo*. Although we have not measured the levels of these chemokines produced from the HD-HIV cells, an increase in their gene expressions of almost over 10 fold indicates their protein levels may also be augmented and may therefore play a crucial role in the development of HIV-1 reservoirs.

Although the levels of productive infection (both p24 protein, *gag *and *Tat *mRNA levels) were almost similar in the HD-HIV and HUT78-HIV cells, there were several other salient differences in the gene expression profiles following HIV-1 infection. In addition to the differences in chemokine and their receptor expressions (Figure 4A), significant differences were seen in several apoptotic markers (Figure 4B) and in several lineage specific transcription factors (Figure 4C). In the HD cells, HIV-1 infection altered the expression of genes associated with apoptosis such as *BAX, BCL2, CASP3 *and *GADD45α*. HD cells also exhibited elevated levels of *BCL11B*, a transcription factor expressed in T-cells [36]. Interestingly, BCL11B has been found to repress HIV-1 transcription from the 5' long terminal repeat [37]. Genes associated with cell cycle regulation, such as *CDKN1A, CDK7 *and most importantly *CDK9*, were also up regulated in the HD-HIV cells, as compared to uninfected HD as well as HUT78-HIV cells. Since, CDK9 plays a crucial role in HIV-1 Tat protein mediated transactivation, a possible role of increased Tat function in the productive infection may also be considered likely. Indeed, the expression of several other transcription factors that are also known to regulate HIV-1 promoter activity, e.g. *CEBP-β *and both *STAT1 *and *STAT3 *genes, were also up regulated in HD-HIV cells, as compared to uninfected HD as well as HUT78-HIV cells. Interestingly, the mRNA expression of *NFκB1A*, the p65 subunit of the transcription factor NFκB which also regulates HIV-1 gene expression in stimulated lymphocytes, was not decisively altered in these cells. However, several cell surface receptors that regulate intracellular NFκB activity, such as TNFSF10 and both IRF1 and IRF2 were higher.

The up-regulation of *Bax*, which results in a loss of mitochondrial membrane polarization and release of pro-apoptotic factors culminating in caspase activation and apoptosis, has been documented [38]. Andersen and coworkers have reported that the expression of *GADD45A *was increased following stressful growth arrest conditions as a result of HIV-1 infection [39]. HIV-1 has also been shown to regulate the expression of *CDK9 *[40]. It has been shown that *STAT3 *promotes the initiation of transcription and regulates chromatin remodeling and transcription elongation through its interaction with *CDK9 *[41].

We also found that the expression of several genes such as *BANF1, BTRC, CD209, APOBEC3F*, and *TAT-SF1 *increased in HD-HIV cells. *BANF1 *is known for its ability to protect retroviruses from intra-molecular integration and there by promoting intermolecular integration into the host cell genome [42]. BTRC interacts with HIV-1 viral protein U (Vpu) and connects CD4 to the proteolytic machinery [43]. *CD209 *expression has been reported in association with HIV-1 infection [44]. APOBEC3F potently restrict HIV-1 replication, and is neutralized by the viral protein Vif [45]. Increased *TAT-SF1 *expression in HD-HIV cells was significant and since it has been shown that *TAT-SF1 *is required for maintaining the ratios of different classes of HIV-1 transcripts [46]. These findings suggest that pathways that facilitate productive infection in T-cells may also be induced in the HD-HIV cells, as is clearly evident from the levels of p24 and *gag *and *Tat *expression in both cell types.

In the present studies for the first time, the infective property of HIV-1 on cells derived from ASCs is reported. It has been reported that HIV-1 stimulates the secretion of the adipocyte-derived hormone adiponectin, however no evidence of infectivity of the virus on adipocytes were shown [47]. Our studies show that ASCs respond to HIV-1 exposure by increasing expression of *IL-10*, *c-Kit*, and *MMD2*. Although these effects do not ultimately result in productive infection, data revealed that HIV-1 exposure increases the hematopoietic lineage commitment of ASCs. The enhanced hematopoietic capacity of HIV-1 exposed ASCs was concurrent with decline in their adipogenic and osteogenic potential. Recently, it has been reported that chronic exposure of CD4^+^, CXCR4^+^, and CCR5^+ ^mesenchymal stem cells with high viral load sera enhanced the adipogenesis [48]. While the treatment of cells with low viral load did not alter differentiation potential of those cells, the ASC clones used in this study were negative for *CD4, CXCR4*, and *CCR5*. In addition, our data suggest no HIV-1 integration into the ASC genome. These results of the present study shed light on the effect of HIV-1 on tissue resident stem cells paving way for additional studies to explore the mechanistic insights for understanding and management of the disease process.

## Conclusion

Based on the observations reported, it is now feasible to study the effect of anti-HIV treatments on ASC derived HD cells. The presence of phenomenal numbers of ASCs in adipose tissue, and these novel findings which indicate that HIV-1 exposure may facilitate their macrophage type commitment, demonstrates that these cells may have importance in generating systemic viral reservoirs. Further, the utility of ASC as well as the ASC derived HD cells as a possible tool for future gene therapy against HIV-1 seems to be promising and merits additional investigation.

## Methods

### Cell culture and Hematopoietic Differentiation

All human tissue sample collection protocols were reviewed and approved by Institutional Review Board (IRB) of Tulane University. Human ASCs were isolated from adipose tissue of healthy donors (n = 14) based on the methods described earlier [49]. ASCs clones were isolated and expanded in α-MEM (CellGro, Manassas, VA) based media, supplemented with 20% fetal bovine serum (Atlanta Biologicals, Lawrenceville, GA), 1% L-Glutamine (CellGro, Manassas, VA) and 1% penicillin/streptomycin (CellGro, Manassas, VA) at 37°C in 5% CO_2_. Then clones were cultured in differentiation media according to a previously described method [25]. Briefly, clonally expanded ASCs were plated at a density of 5000 cells/cm^2 ^on either cell culture dishes or chamber slides (Nalgene, Nunc, Rochester, NY). The differentiation media consisted of α-MEM, 10% FBS, 0.1 μl/ml 1-monothioglycerol (MTG) (Sigma-Aldrich Inc. St. Louis, MO), supplemented with 100 U/ml IL-1ß, 500 U/ml IL-3, and 20 U/ml M-CSF (Prospec Bio, Rehovot, Isreal) as stimulating substances. 30% of the primary volume was augmented with fresh media every 2 days for 12 days. Cultures of ASC clones in growth media containing 10% FBS served as control undifferentiated cells.

### HIV-1 Infection

The uninfected T4-lymphocyte line HUT78, and HUT78 cells persistently infected with HTLV-III_B _strain of HIV-1 (from the AIDS Research & Reference Reagent Program, Bethesda, MD) were cultured in RPMI medium, supplemented with 10% FBS and antibiotics (penicillin & streptomycin). Cell-free viral stocks were obtained from the supernatants of HTLV-III_B _infected cell line grown to 50-60% confluency. The viral titers were determined by measuring HIV-1 p24 levels using an ELISA kit as per the manufacturer's protocol (ZeptoMetrix, Buffalo, NY). For ASC infection studies, cells were cultured in differentiation media for either 5 (5-HD) or 8 (8-HD) days, and subsequently exposed to cell free virus for 24 hr. For HUT-78 cell infection, uninfected cells growing in the logarithmic phase were exposed to cell free virus for 24 hrs. All HIV-1 exposure studies were performed using a viral stock of ~100 pg/ml of p24 [10^3^-10^4 ^transducing units (TU)/ml]. Each viral stock was freshly prepared before exposure of ASCs or uninfected HUT78 cells. For controls, un-differentiated ASCs and HUT78 cells were exposed to the same number of viral particles. Following 24 hrs of virus exposure, cells were washed several times using fresh media to remove the unattached viral particles and cultured for 3 or 5 days post exposure. Prior to viral infection, ASCs were cultured in differentiation media for either 5 or 8 days, and subsequently exposed to HIV-1 in cell free viral media. Viral p24 levels were analyzed at each time point to monitor the viral replication in un-differentiated, HD, and HUT78 cells. A graphical representation of p24 level (pg/ml) vs time point (days) was carried out. Values with p < 0.0001 were considered significant.

### Alu-gag PCR

The genomic DNA from exposed HIV-1 ASCs was subjected to two step *Alu-gag *PCR technique described by Liszewski *et al*. [29]. In the first step the *Alu-gag *regions were amplified using following primers: 1. *Alu *(Forward): 5' GCC TCC CAA AGT GCT GGG ATT ACA G-3'; HIV *gag *(Reverse): nucleotides (nt) 1505-1486 5' GTT CCT GCT ATG TCA CTT CC-3'. On the second step, RU5 region in *gag *was detected using the following primers: RU5 (R Forward): nt 518-539 5'-TTA AGC CTC AAT AAA GCT TGC C-3'; RU5 (U5 Reverse): nt 647-628 5'-GTT CGG GCG CCA CTG CTA GA-3'; 5. RU5wildtype Probe: nt 584-559 5'-CCA GAG TCA CAC AAC AGA CGG GCA CA-3'; RU5degenerate1 Probe: nt 584-559 5'-CCA GAG TCA CAT AAC AGA CGG GCA CA-3'; and RU5degenerate2 Probe: nt 584-559 5'-CCA GAG TCA CAC AAC AGA TGG GCA CA-3'. The PCR products were analyzed by agarose gel electrophoresis.

### RT^2 ^qPCR gene expression analysis

Using total cellular RNA the gene expression was carried out on PCR array kits (SABiosciences, Frederick, MD) which profiles the expression of 84 genes involved in susceptibility to HIV-1, infection and related immune response. The cellular RNAs from un-differentiated ASCs, HD, and HIV-1 infected HD cells (HD-HIV) (n = 3 donors) with HIV-1 infected HUT78 (HUT78-HIV) (serving as positive controls) were used. Data were analyzed using software provided by SABiosciences http://www.sabiosciences.com. Differential gene expression was evaluated for statistical significance (p < 0.05). A cut off of 2 for fold change for up-regulated and 0.5 for down regulated genes was applied, so as to only consider genes whose expression was perturbed in magnitude as well as in a significant manner.

### RT-PCR and Real-Time RT-PCR

Real-Time RT-PCR was performed using SYBR Green Master mix (Invitrogen, Carlsbad, CA) in a 2-step protocol (50 cycles of 10 sec at 90°C and 45 sec at Tm). The following primers were used to assess the gene expressions. *CD4*: 5'-GTA GTA GCC CCT CAG TGC AA-3', 5'-AAA GCT AGC ACC ACG ATG TC-3'; *CD14*: 5'-ACA GGA CTT GCA CTT TCC AG-3', 5'-TCC AGG ATT GTC AGA CAG GT-3'; *CD68*: 5'-CAA CTG CCA CTC ACA GTC CT-3', 5'-CAA TGG TCT CCT TGG AGG TT-3'; *IL10*: 5'-AAG CCT GAC CAC GCT TTC TA-3', 5'-ATG AAG TGG TTG GGG AAT GA-3'; *ITGAM*: 5'-ACG GAT GGA GAA AAG TTT GG-3', 5'-CAA AGA TCT TCT CCC GAA GC-3'; *c-KIT*: 5'-CCG TGG TAG ACC ATT CTG TG-3', 5'-GTG CCC ACT ATC CTG GAG TT-3'; *MMD2*: 5'-GCA GAC CAA GGT GTC CAA AT-3', 5'-CTG GCT GTC ACC AGA AGT CA-3'; *MRC1*: 5'-GGC GGT GAC CTC ACA AGT AT-3', 5'-ACG AAG CCA TTT GGT AAA CG-3'; *MSR1*: 5'-TCC TCG TGT TTG CAG TTC TC-3', 5'-CAT GTT GCT CAT GTG TTC CA-3'; *TNF*: 5'-TCC TTC AGA CAC CCT CAA CC-3', 5'-AGG CCC CAG TTT GAA TTC TT-3'; *gag*: 5'-ATA ATC CAC CTA TCC CAG TAG GAG AAA T-3', 5'-TTT GGT CCT TGT CTT ATG TCC AGA ATG C-3'; *Tat: *5'-GGA ATT CAC CAT GGA GCC AGT AGA TCC T-3', 5'-CGG GAT CCC TAT TCC TTC GGG CCT GT-3'; *GAPDH *5'-CGA GAT CCC TCCA AAA TCA A-3' and 5'-GGT GCT AAG CAG TTG GTG GT-3'. The data were generated using an iCycler MyiQ (Biorad) and analyzed using the iQ5 V2.0 (Bio-Rad). The RT-PCR products were analyzed using agarose gel electrophoresis (1% agarose gel) and stained in 10 μg/ml ethidium bromid (Sigma) for visualization. For real-time RT-PCR, the equation 2^-ΔΔCT ^was used for calculating fold changes. A threshold cycle of 35 was chosen as the cut-off for non-detectable genes, thus genes with CT values above 35 were considered not expressed.

### Immunocytochemistry

HD cells were prepared and infected with HIV, the fixed, permeabilized, and incubated with human specific primary antibodies for CCR4, CCR5, CXCR4, and NOS2 at a final concentration of 0.02-0.04 mg/ml, then incubated with 0.002 mg/ml of the matching secondary antibody. The signal was detected with a Leica TCS SP-2 confocal microscope equipped with Argon (457-477 nm; 488 nm, 514 nm) and HeNe lasers (543 nm; 633 nm) at a magnification of HCX PL APO 63×/1.4 at 21°C. Data were processed with Leica confocal software.

### Osteogenic and Adipogenic Differentiation

Adipogenic differentiation was determined in cultures of ASCs following HIV exposure using previously described methods [16]. Adipogenic potentials were evaluated by oil red O staining. Osteogenic differentiation was induced as previously described [50]. Differentiated cells were either fixed and stained with Alizarin Red (Diagnostic BioSystems) or quantified for alkaline phosphatase activity (ALP) using the SensoLyte™ pNPP Alkaline Phosphatase Assay Kit (AnaSpec, San Jose, CA). All analyzes were carried out in triplicates.

### Statistical analysis

All data relating to this study were summarized using descriptive statistics such as mean, standard deviation and standard error. The analysis of variance method was used to compare the mean differences. Where meaningful, the results were presented graphically. The study hypotheses were tested at 5% level of significance throughout the analysis. Estimates of means and their 95% confidence intervals were calculated. R-computing software was used to plot the graphs.

## Abbreviations

MSCs: mesenchymal stem cells; ASCs: adipose tissue derived mesenchymal stem cells; HD: hematopoietic differentiated cells; AIDS: acquired immune deficiency syndrome; HAART: highly active anti-retroviral therapy; HPCs: hematopoietic progenitor cells; LTBMC: long-term bone marrow cultures; HD-5: differentiate into HD cells for 5 days; HD-8: differentiate into HD cells for 8 days; MOI: multiplicity of infection; HD-HIV: infected HD cells with HIV-1; HUT78-HIV: infected HUT78 cells with HIV-1; ASCs-HIV: exposed ASCs to HIV-1; TRIM5: tripartite motif-containing 5; TAT-SF1: Tat specific factor 1; BTRC: b-transducin repeat containing.

## Competing interests

The authors declare that they have no competing interests.

## Authors' contributions

EF was responsible to cell cloning and cultures. EF, TN, and CS conducted differentiations. UR and CB were responsible for HIV-1 infection studies. AC and CD were responsible for tissue collections. RI, DM, and EA were responsible for experimental design. RI and EA were responsible for the overall experimental design and implementation of the project and contributed equally to this work.

## References

[B1] PerelsonASEssungerPHoDDDynamics of HIV-1 and CD4+ lymphocytes in vivoAIDS199711Suppl AS17249451962

[B2] OggGSJinXBonhoefferSMossPNowakMAMonardSSegalJPCaoYRowland-JonesSLHurleyAMarkowitzMHoDDMcMichaelAJNixonDFDecay kinetics of human immunodeficiency virus-specific effector cytotoxic T lymphocytes after combination antiretroviral therapyJ Virol19997379780010.1128/jvi.73.1.797-800.1999PMC1038929847391

[B3] MooreJPKitchenSGPugachPZackJAThe CCR5 and CXCR4 coreceptors--central to understanding the transmission and pathogenesis of human immunodeficiency virus type 1 infectionAIDS Res Hum Retroviruses20042011112610.1089/08892220432274956715000703

[B4] ZaitsevaMPedenKGoldingHHIV coreceptors: role of structure, posttranslational modifications, and internalization in viral-cell fusion and as targets for entry inhibitorsBiochim Biophys Acta20031614516110.1016/s0005-2736(03)00162-712873765

[B5] RuizMECicalaCArthosJKinterACatanzaroATAdelsbergerJHolmesKLCohenOJFauciASPeripheral blood-derived CD34+ progenitor cells: CXC chemokine receptor 4 and CC chemokine receptor 5 expression and infection by HIVJ Immunol1998161416941769780190

[B6] ChelucciCCasellaIFedericoMTestaUMacioceGPelosiEGuerrieroRMarianiGGiampaoloAHassanHJPeschleCLineage-specific expression of human immunodeficiency virus (HIV) receptor/coreceptors in differentiating hematopoietic precursors: correlation with susceptibility to T- and M-tropic HIV and chemokine-mediated HIV resistanceBlood1999941590160010477684

[B7] BagnaraGPZauliGGiovanniniMReMCFurliniGLa PlacaMEarly loss of circulating hemopoietic progenitors in HIV-1-infected subjectsExp Hematol1990184264301970962

[B8] ReMCZauliGGibelliniDFurliniGRamazzottiEMonariPRanieriSCapitaniSLa PlacaMUninfected haematopoietic progenitor (CD34+) cells purified from the bone marrow of AIDS patients are committed to apoptotic cell death in cultureAIDS199371049105510.1097/00002030-199308000-000047691085

[B9] KokaPSJamiesonBDBrooksDGZackJAHuman immunodeficiency virus type 1-induced hematopoietic inhibition is independent of productive infection of progenitor cells in vivoJ Virol1999739089909710.1128/jvi.73.11.9089-9097.1999PMC11294110516015

[B10] NealTFHollandHKBaumCMVillingerFAnsariAASaralRWingardJRFlemingWHCD34+ progenitor cells from asymptomatic patients are not a major reservoir for human immunodeficiency virus-1Blood199586174917567544640

[B11] GuilakFLottKEAwadHACaoQHicokKCFermorBGimbleJMClonal analysis of the differentiation potential of human adipose-derived adult stem cellsJ Cell Physiol200620622923710.1002/jcp.2046316021633

[B12] FukudaKReprogramming of bone marrow mesenchymal stem cells into cardiomyocytesC R Biol20023251027103810.1016/s1631-0691(02)01524-x12494500

[B13] ZukPAZhuMAshjianPDe UgarteDAHuangJIMizunoHAlfonsoZCFraserJKBenhaimPHedrickMHHuman adipose tissue is a source of multipotent stem cellsMol Biol Cell2002134279429510.1091/mbc.E02-02-0105PMC13863312475952

[B14] WoodburyDReynoldsKBlackIBAdult bone marrow stromal stem cells express germline, ectodermal, endodermal, and mesodermal genes prior to neurogenesisJ Neurosci Res20026990891710.1002/jnr.1036512205683

[B15] TomaCPittengerMFCahillKSByrneBJKesslerPDHuman mesenchymal stem cells differentiate to a cardiomyocyte phenotype in the adult murine heartCirculation2002105939810.1161/hc0102.10144211772882

[B16] IzadpanahRTryggCPatelBKriedtCDufourJGimbleJMBunnellBABiologic properties of mesenchymal stem cells derived from bone marrow and adipose tissueJ Cell Biochem20069912859710.1002/jcb.20904PMC404874216795045

[B17] CanqueBMarandinARosenzwajgMLouacheFVainchenkerWGluckmanJCSusceptibility of human bone marrow stromal cells to human immunodeficiency virus (HIV)Virology199520877978310.1006/viro.1995.12117747451

[B18] ScaddenDTZeiraMWoonAWangZSchieveLIkeuchiKLimBGroopmanJEHuman immunodeficiency virus infection of human bone marrow stromal fibroblastsBlood1990763173221695109

[B19] MosesAVWilliamsSHeneveldMLStrussenbergJRarickMLovelessMBagbyGNelsonJAHuman immunodeficiency virus infection of bone marrow endothelium reduces induction of stromal hematopoietic growth factorsBlood1996879199258562963

[B20] GillVShattockRJScopesJHayesPFreedmanARGriffinGEGordon-SmithECGibsonFMHuman immunodeficiency virus infection impairs hemopoiesis in long-term bone marrow cultures: nonreversal by nucleoside analoguesJ Infect Dis19971761510151610.1086/5141499395362

[B21] SloandEMYoungNSSatoTKumarPKimSWeicholdFFMaciejewskiJPSecondary colony formation after long-term bone marrow culture using peripheral blood and bone marrow of HIV-infected patientsAIDS1997111547155310.1097/00002030-199713000-000029365758

[B22] BahnerIKearnsKCoutinhoSLeonardEHKohnDBInfection of human marrow stroma by human immunodeficiency virus-1 (HIV-1) is both required and sufficient for HIV-1-induced hematopoietic suppression in vitro: demonstration by gene modification of primary human stromaBlood199790178717989292511

[B23] WangLMondalDLa RussaVFAgrawalKCSuppression of clonogenic potential of human bone marrow mesenchymal stem cells by HIV type 1: putative role of HIV type 1 tat protein and inflammatory cytokinesAIDS Res Hum Retroviruses20021891793110.1089/08892220276026559712230935

[B24] LawrenceDMDurhamLCSchwartzLSethPMaricDMajorEOHuman immunodeficiency virus type 1 infection of human brain-derived progenitor cellsJ Virol2004787319732810.1128/JVI.78.14.7319-7328.2004PMC43411115220405

[B25] FreisingerECramerCXiaXMurthySNSlakeyDPChiuENewsomeERAltEUIzadpanahRCharacterization of hematopoietic potential of mesenchymal stem cellsJ Cell Physiol20102258889710.1002/jcp.2229920635396

[B26] GorryPRChurchillMCroweSMCunninghamALGabuzdaDPathogenesis of macrophage tropic HIV-1Curr HIV Res20053536010.2174/157016205277295115638723

[B27] KedzierskaKCroweSMThe role of monocytes and macrophages in the pathogenesis of HIV-1 infectionCurr Med Chem200291893190310.2174/092986702336893512369874

[B28] CassolEAlfanoMBiswasPPoliGMonocyte-derived macrophages and myeloid cell lines as targets of HIV-1 replication and persistenceJ Leukoc Biol2006801018103010.1189/jlb.030615016946020

[B29] LiszewskiMKYuJJO'DohertyUDetecting HIV-1 integration by repetitive-sampling Alu-gag PCRMethods20094725426010.1016/j.ymeth.2009.01.002PMC286246919195495

[B30] AndersonJSBandiSKaufmanDSAkkinaRDerivation of normal macrophages from human embryonic stem (hES) cells for applications in HIV gene therapyRetrovirology200632410.1186/1742-4690-3-24PMC146299716623949

[B31] GibelliniDReMCVitoneFRizzoNMaldiniCLa PlacaMZauliGSelective up-regulation of functional CXCR4 expression in erythroid cells by HIV-1 Tat proteinClin Exp Immunol200313142843510.1046/j.1365-2249.2003.02095.xPMC180866012605695

[B32] XiaoHNeuveutCTiffanyHLBenkiraneMRichEAMurphyPMJeangKTSelective CXCR4 antagonism by Tat: implications for in vivo expansion of coreceptor use by HIV-1Proc Natl Acad Sci USA200097114661147110.1073/pnas.97.21.11466PMC1722311027346

[B33] MondalDWilliamsCAAliMEilersMAgrawalKCThe HIV-1 Tat protein selectively enhances CXCR4 and inhibits CCR5 expression in megakaryocytic K562 cellsExp Biol Med (Maywood)200523063164410.1177/15353702052300090516179731

[B34] CocchiFDeVicoALGarzino-DemoAAryaSKGalloRCLussoPIdentification of RANTES, MIP-1 alpha, and MIP-1 beta as the major HIV-suppressive factors produced by CD8+ T cellsScience19952701811181510.1126/science.270.5243.18118525373

[B35] MajkaMRozmyslowiczTLeeBMurphySLPietrzkowskiZGaultonGNSilbersteinLRatajczakMZBone marrow CD34(+) cells and megakaryoblasts secrete beta-chemokines that block infection of hematopoietic cells by M-tropic R5 HIVJ Clin Invest19991041739174910.1172/JCI7779PMC40988210606628

[B36] LiPBurkeSWangJChenXOrtizMLeeSCLuDCamposLGouldingDNgBLDouganGHuntlyBGottgensBJenkinsNACopelandNGColucciFLiuPReprogramming of T Cells to Natural Killer-Like Cells upon Bcl11b DeletionScience201032985910.1126/science.1188063PMC362845220538915

[B37] MarbanCSuzanneSDequiedtFde WalqueSRedelLVan LintCAunisDRohrORecruitment of chromatin-modifying enzymes by CTIP2 promotes HIV-1 transcriptional silencingEMBO J20072641242310.1038/sj.emboj.7601516PMC178344917245431

[B38] MuthumaniKChooAYPremkumarAHwangDSThieuKPDesaiBMWeinerDBHuman immunodeficiency virus type 1 (HIV-1) Vpr-regulated cell death: insights into mechanismCell Death Differ200512Suppl 196297010.1038/sj.cdd.440158315832179

[B39] AndersenJLZimmermanESDeHartJLMuralaSArdonOBlackettJChenJPlanellesVATR and GADD45alpha mediate HIV-1 Vpr-induced apoptosisCell Death Differ20051232633410.1038/sj.cdd.440156515650754

[B40] SedoreSCByersSABiglioneSPriceJPMauryWJPriceDHManipulation of P-TEFb control machinery by HIV: recruitment of P-TEFb from the large form by Tat and binding of HEXIM1 to TARNucleic Acids Res2007354347435810.1093/nar/gkm443PMC193500117576689

[B41] GiraudSHurlstoneAAvrilSCoqueretOImplication of BRG1 and cdk9 in the STAT3-mediated activation of the p21waf1 geneOncogene2004237391739810.1038/sj.onc.120797215286705

[B42] MansharamaniMGrahamDRMonieDLeeKKHildrethJESilicianoRFWilsonKLBarrier-to-autointegration factor BAF binds p55 Gag and matrix and is a host component of human immunodeficiency virus type 1 virionsJ Virol200377130841309210.1128/JVI.77.24.13084-13092.2003PMC29606714645565

[B43] ChristodoulopoulosIDroniou-BonzomMEOldenburgJECannonPMVpu-dependent block to incorporation of GaLV Env into lentiviral vectorsRetrovirology20107410.1186/1742-4690-7-4PMC283100820102634

[B44] Serrano-GomezDSierra-FilardiEMartinez-NunezRTCaparrosEDelgadoRMunoz-FernandezMAAbadMAJimenez-BarberoJLealMCorbiALStructural requirements for multimerization of the pathogen receptor dendritic cell-specific ICAM3-grabbing non-integrin (CD209) on the cell surfaceJ Biol Chem20082833889390310.1074/jbc.M70600420018073208

[B45] DangYDavisRWYorkIAZhengYHIdentification of 81LGxGxxIxW89 and 171EDRW174 domains from human immunodeficiency virus type 1 Vif that regulate APOBEC3G and APOBEC3F neutralizing activityJ Virol2010845741575010.1128/JVI.00079-10PMC287661020335268

[B46] MillerHBSaundersKOTomarasGDGarcia-BlancoMATat-SF1 is not required for Tat transactivation but does regulate the relative levels of unspliced and spliced HIV-1 RNAsPLoS One20094e571010.1371/journal.pone.0005710PMC268265819479034

[B47] SankaleJLTongQHadiganCMTanGGrinspoonSKKankiPJHotamisligilGSRegulation of adiponectin in adipocytes upon exposure to HIV-1HIV Med2006726827410.1111/j.1468-1293.2006.00372.x16630040

[B48] CotterEJChewNPowderlyWGDoranPPHIV Type 1 Alters Mesenchymal Stem Cell Differentiation Potential and Cell Phenotype ex VivoAIDS Res Hum Retroviruses2010 in press 10.1089/aid.2010.011420929345

[B49] ZukPAZhuMMizunoHHuangJFutrellJWKatzAJBenhaimPLorenzHPHedrickMHMultilineage cells from human adipose tissue: implications for cell-based therapiesTissue Eng2001721122810.1089/10763270130006285911304456

[B50] IzadpanahRJoswigTTsienFDufourJKirijanJCBunnellBACharacterization of multipotent mesenchymal stem cells from the bone marrow of rhesus macaquesStem Cells Dev20051444045110.1089/scd.2005.14.44016137233

